RETRACTED

# The Potential Function of Super Enhancers in Human Bone Marrow Mesenchymal Stem Cells during Osteogenic Differentiation

**DOI:** 10.1155/2021/6614762

**Published:** 2021-01-26

**Authors:** Zhijie Huang, Bo Jia, Qian Wang, Naishun Wang, Jianjiang Zhao

**Affiliations:** ^1^Departments of Oral and Maxillofacial Surgery, Stomatological Hospital, Southern Medical University (Guangdong Provincial Stomatological Hospital), Guangzhou, Guangdong 510280, China; ^2^Department of Central Laboratory, Taian Central Hospital, Longtan Road No. 29, Tai'an, 271000 Shandong Province, China; ^3^Department of Orthopaedics, Taian Hospital of Traditional Chinese Medicine, Yingxuan Street No. 216, Taishan District, Tai'an, 271000 Shandong Province, China; ^4^Departments of Oral and Maxillofacial Surgery, Shenzhen Stomatological Hospital, Southern Medical University (Shenzhen Dental Medical Center of Guangdong Province), Shenzhen, Guangdong 518001, China

## Abstract

Super enhancers (SEs) are large clusters of transcriptional activity enhancers, which drive and control the expression of cell identity genes, as well as differentiation of specific cell types. SEs have great application potential in pathogenic mechanism studies in developmental biology, cancer, and other diseases. However, the potential function and regulatory mechanism of SEs in the osteogenic differentiation of human bone marrow mesenchymal stem cells (hBMSCs) are unknown. Therefore, this study investigated the potential function of SEs in the osteogenic differentiation of hBMSCs and their target genes. Osteogenesis was induced in three hBMSCs groups for 14 days. Further, ChIP-seq was performed on cells before and after osteogenic differentiation. Two target genes were then selected from cells before and after osteogenic differentiation for RT-qPCR. Finally, the selected SE target genes were analyzed by bioinformatics. In total, 1,680 SEs were identified in hBMSCs. After 14 days of osteogenic induction, only 342 SEs were detected in cells, among which 1,380 unique SEs were detected in hBMSCs, 42 unique SEs were found in cells induced by osteoblast differentiation after 14 days, and 300 SEs were common in both groups. Further, 1,680 genes were found to be regulated by SEs in hBMSCs, including 1,094 genes with protein-coding function and 586 noncoding genes. Additionally, 342 genes were regulated by SEs in cells after 14 days of osteogenic differentiation induction, of which 223 and 119 had protein-coding and noncoding functions, respectively. KEGG analysis of SE target genes before and after osteogenic differentiation showed the TGF-*β*, PI3K-Akt, and ECM receptor signaling pathways as highly enriched and closely related to osteogenic differentiation. Further, RT-qPCR results of four selected target genes confirmed the sequencing results. Taken together, osteogenic differentiation of hBMSCs involves changes in multiple SEs, which may regulate the osteogenic differentiation of hBMSCs by regulating the expression of target genes.

RETRACTED

## 1. Introduction

The maxillofacial bone defect is often caused by trauma, infection, congenital malformation, or cancer surgery, which not only affects the facial aesthetic, as well as mastication and swallowing functions, but also often results in psychological and social challenges for patients [1]. Due to the complex structure of the maxillofacial bone, repairing defects often pose significant challenges. Currently, bone transplantation is a common clinical practice with autologous bone transplantation considered the “gold standard” for bone transplantation; however, this procedure has numerous adherent disadvantages, including damage to the donor site, limited available bone, and poor bone quality in patients with osteoporosis and other diseases [2]. Although synthetic bone can be used to replace autologous bone, specific limitations often arise, including immunogenicity, risk of infection, low bone induction, and poor bone integration [3]. Alternatively, bone tissue engineering techniques combine stem cells with biological scaffold materials to form reconstructed tissue with similar functional characteristics to natural bone tissue through specific bone inducing factor stimulation. This strategy is expected to become a novel method for bone repair soon [4] and consists of the following components: seed cells (most critical), growth factors, and biological scaffold materials. Human bone marrow mesenchymal stem cells (hBMSCs) are a diverse group of cells with multidirectional differentiation potential. When tissues or cells in the body are stimulated by the local microenvironment during periods of tissue damage or disease, they become stimulated to release cytokines, growth factors, etc., thus stimulating BMSCs to differentiate into various connective tissue cells, including articular cartilage, bone, muscle, and tendon tissues. In addition, these cells can be amplified and cultured *in vitro* or *in vivo* to ultimately differentiate into osteoblasts, chondrocytes, fat cells, tendon cells, muscle tubes, and nerve cells, among others [5]. Therefore, BMSCs are often employed as seed cells for bone tissue engineering. Hence, further investigation into the currently uncharacterized osteogenic differentiation mechanism of BMSCs may serve to promote the application of bone tissue engineering in clinical practice.

Super enhancers (SEs) are a large cluster of transcriptional enhancers [6] that span, by order of magnitude, more DNA than typical enhancers (TEs). In addition, many cell-specific master transcription factor-binding motifs are enriched in SEs, enabling SEs to bind to a larger number of transcription factors, cofactors, and transcriptional activity-related histone modification markers with higher density. Further, these characteristics provide SEs with stronger transcriptional activation activity and higher interference sensitivity, which can drive and control the expression of cell identity genes, as well as regulate specific expression patterns in different cell types, thereby offering great application potential in developmental biology research related to the pathogenic mechanisms in cancer and other diseases [6, 7]. However, the potential function and molecular mechanism of SEs in osteogenic differentiation of hBMSCs are not characterized yet.

RETRACTED

In this study, osteogenic differentiation of three hBMSCs groups was carried out, and ChIP-seq was performed on cells before and after osteogenic differentiation in order to screen and identify SEs related to osteogenic differentiation of hBMSCs. Further, bioinformatics analysis was conducted for their target genes to predict their potential functions in osteogenic differentiation, laying the foundation for further investigations on the osteogenic differentiation of hBMSCs, and providing new regulatory targets for the construction of novel tissue-engineered bone grafts.

## 2. Materials and Methods

### 2.1. Culture and Osteogenic Differentiation of hBMSCs

Frozen primary hBMSCs (Saliai, Guangzhou, China) were rapidly placed in a water bath at 37°C until thawed. The primary hBMSCs were inoculated at a density of 5 × 10^3^/cm^2^ in a T-25 culture flask and cultured at 37°C in 5% CO_2_. Once the cells reached 90–95% confluence, they were transferred to and cultured on 6-well plates. The cells were then divided into two groups: culture without treatment (D0 group) and culture with osteoblastic differentiation fluid treatment (Cyagen, Suzhou, China, HUXMA-90021), according to the manufacturer's instructions (D14 group). The culture medium was replaced every three days, and cells were collected after 14 days of culture.

### 2.2. Alizarin Red Staining

The culture medium for the D0 and D14 groups was absorbed and washed with PBS three times. Cells were fixed with 4% paraformaldehyde at 25°C for 30 min and rinsed with distilled water thrice. The cells were then stained with 0.1% alizarin red for 30 min at 37°C. Subsequently, the cells were washed with distilled water, dried, and observed under a microscope (Aote, Chongqing, China, BDS200-FL). Finally, the images were collected and analyzed.

RETRACTED

### 2.3. RNA Extraction and RT-qPCR

Total RNA was extracted from D0 and D14 cells using the TRIzol kit (MRC, Ohio, USA, TR118-500) according to the manufacturer's instructions. The quality of the total RNA extracted was measured. The PCR reaction system was performed according to protocols provided with the qPCR detection kit (Vazyme, Nanjing, China, Q341-03). The initial activation of the qPCR reaction was conducted at 95°C for 120 s, and subsequently, 40 cycles were performed at the following settings: denaturation, 95°C, 30 s; annealing, 60°C, 30 s; extension, 72°C, 45 s. A final extension was performed at 75°C for 4 min and repeated thrice. *GAPDH* was used as an internal reference gene. After the qPCR reaction, Ct values of the target gene and internal reference gene were obtained through the real-time fluorescence curve. Finally, mRNA expression levels in the D0 and D14 groups were analyzed by 2^-*ΔΔ*Ct^. The primers for *RUNX2*, *OPN*, *COL1A1*, and *GAPDH* are provided in Table 1.

### 2.4. Western Blot

After osteogenic induction, cells were collected and lysed with RIPA buffer (Beyotime, Shanghai, China) to obtain total protein content. Protein levels were quantified using the Bradford kit (Pierce, Illinois, USA) and electrophoresis on a 10% SDS-polyacrylamide gradient gel. The proteins were then transferred to a polyvinylidene fluoride membrane (Millipore, Massachusetts, USA) and incubated in 5% bovine serum albumin for one hour. Further, protein expression was detected using anti-RUNX2 (CST, Massachusetts, USA, diluted 1 : 2,000), anti-OPN (Abcam, Cambridge, UK, diluted 1 : 2,000), and anti-COL1A1 (Abcam, diluted 1 : 2,000) antibodies. Antibody diluent was added to the membrane and incubated overnight at 4°C. Subsequently, the membranes were incubated at room temperature with secondary enzyme-labeled antibodies (Abcam, ab6721, 1 : 2,000 dilution) for one hour. HRP signals were detected using a chemiluminescence reagent (Millipore). Protein expression was quantified using the BCA protein quantification method and was normalized against GAPDH (Abcam, diluted 1 : 500). The ImageJ software (National Institutes of Health, Bethesda, MD, USA) was used to process the image.

### 2.5. Chromatin Immunoprecipitation-Sequencing (ChIP-seq)

In brief, 8 × 10^6^ fresh cells were extracted and suspended in 10 mL medium. Chromatin immunoprecipitation was performed using the EpiTM chromatin immunoprecipitation kit (Epibiotek, Guangzhou, China, cat. no. R1802) according to the manufacturer's instructions. Cells were harvested and cross-linked with 1% formaldehyde for 10 min, followed by quenching with 0.125 M glycine for 5 min. Cells were lysed in 1 mL lysis buffer and rotated for 30 min at 4°C. Further, cell lysates were centrifuged at 2,400 × *g* for 10 min at 4°C to isolate the nuclei. The nuclei were suspended in digestion buffer and subjected to enzymatic shearing to generate 200–500 bp chromatin fragments at 37°C for 10–15 min. Next, the shearing reaction was stopped, and the fragmented chromatin was centrifuged at 18,000 × *g* for 10 min at 4°C. The supernatant was transferred to a new Eppendorf tube, and the chip reaction mix was added containing protein A/G magnetic beads, chip IP buffer, antibodies, and protease inhibitor cocktail and rotated at 4°C overnight. Protein A/G magnetic beads were then washed. The chromatin was eluted in the reverse cross-linking buffer, followed by incubation at 65°C for 3 h. Subsequently, the ChIP DNA was treated with RNase A and protease K at 37°C for 30 min and purified using Phenol chloroform. ChIP DNA was processed for library generation using the QIAseq Ultralow Input Library Kit (QIAGEN, Hilden, Germany) following the manufacturer's protocol.

RETRACTED

### 2.6. Identification of Super Enhancers

ChIP-seq reads were aligned to the human reference genome by Bowtie Aligner [8]. ChIP-seq reads aligning to the region were extended by 200 bp, and the density of reads per base pair (bp) was calculated. The density of reads in each region was normalized to the total number of million mapped reads, producing read density in units of reads per million mapped reads per base pair (rpm/bp). ChIP-seq peaks were identified using MACS (Model-Based Analysis of ChIP-seq) by considering reads mapped only once at a given locus. Enhancers were defined as regions of ChIP-seq enrichment for H3K27ac. Closely spaced peaks within a range of 12.5 kb were merged together, followed by measurement of input and H3K27ac signals. These merged peaks were ranked by H3K27ac signal and then classified as SEs or TEs [6].

### 2.7. Functional Enrichment Analysis

According to the location of the SE, target genes were predicted, and the functions and pathways of these genes were analyzed through multiple databases. GO (Gene Ontology) analysis was conducted using the DAVID database (Database for Annotation, Visualization, and Integrated Discovery; http://david.abcc.ncifcrf.gov/), in which the molecular function of target genes can be determined. The default algorithm of the database (Fisher's exact test) was used to obtain *P* values related to GO term enrichment, and *P* < 0.05 was considered statistically significant. KEGG (Kyoto Encyclopedia of Gene and Pathway Analysis) analysis (KEGG biological pathway database; http://www.genome.jp/) was used to identify biological pathways associated with target genes. Using the default algorithm in the database (Fisher's exact test), *P* values related to the enrichment of SE target genes in each biological pathway were obtained. *P* < 0.05 was considered statistically significant.

RETRACTED

### 2.8. Validation of SE Target Gene Expression

Two target genes were selected from the D0 and D14 groups to verify the accuracy of sequencing results. The RT-qPCR method has been described previously. The target genes and their primers are provided in Table 2.

### 2.9. Statistical Analysis

The SPSS13.0 software was used for statistical analysis, and measurement data were expressed as mean ± standard deviation. Two independent sample Student's *t*-tests were conducted. In addition, one-way ANOVA and post hoc Student-Newman-Keuls test were used for comparison between groups. *P* < 0.05 was considered statistically significant.

## 3. Results

### 3.1. Osteogenic Differentiation of hBMSCs

After culturing primary hBMSCs to P2 generation, the cells exhibited long spindle morphology and unique growth characteristics. After 14 days of osteogenic induction and culture, the cells began to aggregate and showed irregular morphology, including primarily polygonal or cubic shapes.

After 14 days of osteogenic induction and differentiation, alizarin red staining showed red calcium deposition nodules (Figure 1(a)). RNA and protein were extracted from hBMSCs before (D0) and 14 days after (D14) osteogenic-induced differentiation. Further, mRNA and protein expression levels of osteogenic-specific transcription factors (RUNX2, OPN, and COL1A1) were detected by qPCR and Western blot, respectively, for which RUNX2, OPN, and COL1A1 mRNA (Table 3, Figure 1(b)) and protein (Table 4, Figures 1(c) and 1(d)) expression levels were significantly higher after 14 days of osteogenic differentiation induction (*P* < 0.05).

### 3.2. Screening of SEs in hBMSCs before and after Osteogenic Differentiation by Chromatin Immunoprecipitation-Sequencing (ChIP-seq)

In total, 31,470 enhancers were identified from the D0 group by the ChIP-seq method, including 1,680 SEs with a cutoff value of 17,825.97 (Figure 2(a), and Table 5). Detailed information is provided in Table 3. In the D14 group, 5,119 enhancers were identified, of which 342 were super-enhancers, with a cutoff value of 2,761.05 (Figure 2(b) and Table 6), among which 300 SEs were shared between the D0 and D14 groups, 1,380 SEs were unique to D0, and 42 SEs were unique to D14. Additionally, the target genes of SEs were analyzed, identifying 1,680 SE target genes in the D0 group, including 1,094 protein-coding and 586 noncoding genes. Further, 342 SE target genes in the D14 group were identified, among which 223 were protein-coding, and 119 were noncoding genes. To validate the sequencing results, two unique SE target genes were selected randomly from the D0 (LINC00460 and LINC00844) and D14 (KCNMA1-AS1 and ASTN2-AS1) groups for RT-qPCR verification. Results showed that relative mRNA expression levels of LINC00460 and LINC00844 after osteogenesis differentiation were significantly decreased compared to expression before differentiation (Table 7, Figure 3(a)), whereas KCNMA1-AS1 and ASTN2-AS1 were significantly increased (Table 7, Figure 3(b)).

RETRACTED

### 3.3. GO and KEGG Biological Pathway Enrichment Analyses

GO analysis was conducted for SE target genes in the D0 and D14 groups, at *P* < 0.05 and an enrichment score of -log (*P* value). For the D0 group, the top three GO terms in BP (biological process) were extracellular matrix organization, axon guidance, and cell adhesion, with 49, 61, and 67 genes, respectively (Figure 4(a)). In CC (cellular component), the top three GO terms were focal adhesion, proteinaceous extracellular matrix, and cytoplasm, with 56, 46, and 398 genes, respectively (Figure 4(a)). For MF (molecular function), the top three enrichment scores were for protein binding, collagen binding, and SH3 domain binding, with 497, 16, and 22 genes, respectively (Figure 4(a)). In the D14 group, the top GO enrichment terms in BP were regulation of interleukin-1*β* secretion, negative regulation of retinal ganglion cell axon guidance, and extracellular matrix disassembly, with 2, 2, and 7 genes, respectively (Figure 4(b)). In CC, the top three GO terms were basement membrane, ruffle, and focal adhesion, with 6, 6, and 12 genes, respectively (Figure 4(b)). In MF, the top three enrichment scores were for proteoglycan binding, peptide hormone binding, and methenyltetrahydrofolate cyclohydrolase activity, with 497, 16, and 22 genes, respectively (Figure 4(b)).

Through KEGG analysis of SE-related target genes in the D0 and D14 groups, at *P* < 0.05 and enrichment score of -log (*P* value), the top three pathways in the D0 group were determined to be proteoglycans in cancer, pathways in cancer, and TGF-*β* signaling pathway, which are closely related to osteogenic differentiation pathways (Figure 5(a)). In the D14 group, the top three pathways were ECM receptor interaction, proteoglycans in cancer, and PI3K-Akt signaling pathway, for which the ECM receptor interaction and PI3K-Akt signaling pathway were closely related to the osteogenic differentiation pathway (Figure 5(b)).

## 4. Discussion

Human bone marrow mesenchymal stem cells have the potential to differentiate into bone, cartilage, fat, nerve, and other tissues. They can be extracted and separated from the autologous bone marrow of patients. As one of the ideal bone tissue engineering seed cells, they have been widely used in the construction of tissue engineering bone [9–11]. Compared with other stem cells, hBMSCs have shown greater advantages in osteogenesis differentiation, self-renewal ability, and secretion of growth factors, cytokines, and chemokines bioactive factors to regulate immune responses and enhance tissue regeneration [12–15]. Therefore, studying the osteogenic differentiation mechanism of hBMSCs will provide an important basis for the clinical application of bone tissue engineering.

RETRACTED

Enhancers are DNA sequences that can significantly increase the frequency of gene transcription and contain multiple transcription factor binding sites. Cells control the transcription process primarily through binding transcription factors that control cell type-specific gene expression patterns [16–18]. SEs were proposed by Young et al. in 2013. They identified enhancers on mouse embryonic stem cells through genomic analysis of master transcription factors (mTFs) and mediator binding sites through ChIP-seq technology. Enhancers are generally divided into typical enhancers (TEs) and SEs based on ChIP-seq signal levels. SEs are rich in cell-specific key transcription factor binding motifs. These structural features enable it to bind to more transcription factors, cofactors, and transcriptional activity-related histone modification markers with higher density. Taken together, these characteristics give SEs stronger transcriptional activation ability and higher interference sensitivity, which drive and control the expression of cell identity genes and determine the specific expression pattern in different cell types, showing great application potential in developmental biology and studies related to pathogenic mechanisms in cancer and other diseases [14, 15].

SEs can regulate cell development and differentiation by driving the expression of cell identity genes. For example, SEs of progenitor B cells can bind to the transcription factor PU.1 at high density and activate transcription of Foxo1 and Inpp5d genes. Foxo1 is involved in determining the phenotype of B lymphocytes [19], whereas Inpp5d is involved in responses to B-cell antigen receptor signals [20]. Muscle tubule cell SE sequences can be combined with transcription factors MyoD, key for promoting transcription of the muscle cytoskeletal protein Myoglobin [21]. In T helper cells, SEs binds to the transcription factor T-bet to regulate Tcf7 gene, which is involved in the formation of T cells in the hematopoietic process [22]. SEs of macrophages are bound to transcription factor C/EBP-*α*, in which its downstream genes encode extracellular matrix glycoproteins, and thus participate in the recognition and clearance of apoptotic cells by macrophages [23]. In the process of preadipocyte early fat synthesis, Med1 and other important transcription factors in highly integrated hot areas (hotspots) constitute the key components of SEs, usually by interfering with hotspots and SE regional combination of transcription factors to control preadipocyte differentiation [24].

RETRACTED

To our knowledge, this study is the first to screen SEs involved in osteogenic differentiation of hBMSCs by ChIP-seq. To validate the sequencing results, four SE-related target genes were selected from cells before and after osteogenic differentiation for RT-qPCR verification. Although a large number of studies have shown that SEs can participate in cell development and differentiation, few studies have focused on osteogenic differentiation of hBMSCs and how SEs regulates osteogenic differentiation through their target genes. Previous research has confirmed that the Wnt/*β*-catenin, p38 mitogen-activated protein kinase (MAPK), Notch signal, nuclear factor-kappa B (NF-*κ*B) signaling, BMP signaling, fibroblast growth factor (FGF) signaling, and ECM signaling pathways play important roles in the osteogenic differentiation process [25, 26]. For example, the Wnt/*β*-catenin pathway is a key regulator of bone homeostasis and one of the most common targets for interventional treatment of fracture patients [27]. It has long been accepted that *β*-catenin can activate osteogenic differentiation and osteogenesis, stimulating osteoblasts to produce osteogenic-specific transcription factors such as Runx2 and Osterix [28]. BMPs belong to the TGF-*β* superfamily, and numerous studies have shown that BMPs bind to receptor complexes consisting of heterotetramers of type I and type II Ser/Thr kinase receptors and activate SMADs (SMAD1, SMAD5, or SMAD8) through site-specific phosphorylation. Subsequently, phosphorylated SMADs form complexes with SMAD4 and enter the nucleus to regulate gene expression, thereby regulating osteogenic differentiation [29]. FGFs are a large family of proteins, most of which act by binding to Tyr kinase FGF receptors on the cell surface, triggering phosphorylation of a series of signaling proteins and activation of multiple signaling modules, including MAPK, phosphoinositide 3-kinase (PI3K), STAT1, and PKC [30]. These pathways are classical osteogenesis signaling pathways through which many target genes participate in the regulation of osteogenesis. In this study, bioinformatics was performed to conduct GO and KEGG analyses on SE target genes to determine the biological functions and pathways related to osteogenic differentiation. The top pathways with the highest enrichment scores in KEGG analysis included TGF-*β*, PI3K-Akt, and ECM receptor signaling pathways, which were closely related to osteogenic differentiation. The TGF-*β* signaling pathway is involved in many cellular processes and has multiple regulatory mechanisms. In the process of osteogenic differentiation of mesenchymal stem cells, TGF-*β* can interact with SMAD and BMP through the TGF-*β* type I receptor, thereby regulating osteogenic differentiation. Further, Li et al. [31] found that upregulation of miRNA-10b could promote osteogenic differentiation of mesenchymal stem cells, while downregulation could inhibit osteogenic differentiation. Target prediction and dual-luciferase reporter gene analysis identified SMAD2 as a potential target for miR-10b, demonstrating that it may regulate the osteogenic differentiation process through TGF-*β* signaling. Huang et al. [32] found that LncRNA H19 regulates osteogenic differentiation of BMSCs through the TGF-*β* signaling pathway. Taken together, all these studies suggest that TGF-*β* signaling pathways play an important role in osteogenic differentiation in mesenchymal stem cells. Therefore, SEs may regulate the osteogenic differentiation of BMSCs by regulating the expression of target genes and, in turn, the TGF-*β* signaling pathway.

RETRACTED

It is worthwhile to acknowledge the significance of the present study and its implications for future research. First, the epigenetic mechanisms that we have researched from the aspect of SE-LncRNAs provided a theoretical basis and a better understanding of the researchers in the area of BMSCs-osteodifferentiation. Second, the SE-LncRNAs biomarkers identified could provide the research directions for future experimental studies regarding the epigenetic mechanisms of BMSCs. Second, since many previous studies have shown that the epigenetic modification of BMSCs can obtain better osteodifferentiation capacity compared with BMSCs without any modification, the SE-LncRNAs identified in this study might be used for the epigenetic modification of BMSCs and further promote the osteogenic ability of BMSCs. The BMSCs with epigenetic manipulation have the potential to be used for the 3D-tissue engineered constructs for the treatment of periodontal defects, peri-implant bone defects, and maxillofacial bone defects in the dental area.

## 5. Conclusions

The current study suggests that SEs play an important role in the osteogenic differentiation of hBMSCs, providing new targets and theoretical basis for bone tissue engineering. Future studies will select 3–5 SE-related target genes for functional verification, to confirm their role in the osteogenic differentiation of hBMSCs, and to verify their mechanisms and pathways.

RETRACTED

## Figures and Tables

**Figure 1:** Identification of osteogenic differentiation of hBMSCs. (a) Alizarin red staining (magnification ×100). (b) Relative mRNA expression levels of osteogenesis-specific transcription factors RUNX2, OPN, and COL1A1, as detected by RT-qPCR. (c, d) Western blot (WB; c) and corresponding quantification (d) of osteogenesis-specific transcription factors RUNX2, OPN, and COL1A1. GAPDH was used as a loading control. ∗∗ indicates *P* < 0.01; ∗∗∗ indicates *P* < 0.001; ∗∗∗∗ indicates *P* < 0.0001.

**Figure 2:** Super-enhancers in BMSCs (D0 group) and osteoblasts (D14 group). (a) Distribution of ChIP-seq density across enhancers with 1680 SEs and a cutoff value of 17825.97 in the D0 group (ranked by H3K27ac signal. (b) Distribution of ChIP-seq density across enhancers with 342 SEs and a cutoff value of 2761.06 in the D14 group (ranked by H3K27ac signal. (c) The comparison of D0 group and D14 group super-enhancers.

**Figure 3:** RT-qPCR validation of SE target genes during BMSC osteogenic differentiation. (a) SE target genes in the D0 group. (b) SE target genes in the D14 group. ∗∗∗ indicates *P* < 0.001; ∗∗∗∗ indicates *P* < 0.0001.

**Figure 4:** Gene ontology analyses of SE target genes. (a) Top 15 enrichment scores for biological processes, cellular components, and molecular functions among SE target genes of the D0 group. (b) Top 15 enrichment scores for biological processes, cellular components, and molecular functions among SE target genes of the D14 group.

**Figure 5:** Kyoto Encyclopedia of Genes and Genomes analyses of SE target genes. (a) Top 15 enriched pathways in KEGG analysis for SE target genes in the D0 group. (b) Top 15 enriched pathways in KEGG analysis for SE target genes in the D14 group.

**Table 1:** Primer sequences used in quantitative polymerase chain reaction validation. Osteogenesis-specific transcription factors.

Primer	Sequence (5'⟶3')
OPN q forward	AGACCCTTCCAAGTAAGTCC
OPN q reverse	TCATCTACATCATCAGAGTCGT
COL1A1 q forward	GCCAAGACGAAGACATCCCA
COL1A1 q reverse	GGCAGTTCTTGGTCTCGTCA
RUNX2 q forward	TGGTTACTGTCATGGCGGGTA
RUNX2 q reverse	TCTCAGATCGTTGAACCTTGCTA

**Table 2:** Primer sequences used in quantitative polymerase chain reaction validation. SE target genes.

Primer	Sequence (5'⟶3')
LINC00460 q forward	TGGATGAACCACCATTGCCA
LINC00460 q reverse	TCGGGGTGACTTCAGAATGC
LINC00884 q forward	TGATTTTCGCTGCGTCCTCT
LINC00884 q reverse	GGCGGCTGAGTTCTGTAAGT
KCNMA1-AS1 q forward	ATGTTCTTCCCAACCTGCCAA
KCNMA1-AS1 q reverse	CTCAAACACGAGCGGACCAG
ASTN2-AS1 q forward	AAGTTGGCACACAGCACTCT
ASTN2-AS1 q reverse	ATTTCTACCTCCCGCTTGCC

RETRACTED

**Table 3:** The RUNX2, OPN, and COL1A1 gene expression change during osteogenesis of hBMSCs.

Osteogenesis-specific transcription factors	D0	D14
RUNX2	1.07 ± 0.07	2.73 ± 0.20
OPN	0.92 ± 0.07	28.77 ± 1.89
COL1A1	0.92 ± 0.06	3.23 ± 0.17

**Table 4:** The RUNX2, OPN, and COL1A1 protein expression change during osteogenesis of hBMSCs.

Osteogenesis-specific transcription factors	D0	D14
RUNX2	0.59 ± 0.01	0.89 ± 0.01
OPN	0.12 ± 0.01	0.85 ± 0.01
COL1A1	0.84 ± 0.01	1.24 ± 0.01

**Table 5:** Detailed information of super enhancers. D0 group.

ID	Chrom	Start	End	Size	Target gene	Gene type
4_BMSC_peak_18504_lociStitched	Chr11	76073282	76088184	14902	WNT11	Protein-coding
25_BMSC_peak_100453_lociStitched	Chr7	82131135	82211994	80859	LOC101927356	ncRNA
3_BMSC_peak_80926_lociStitched	Chr5	31360700	31378910	18210	DROSHA	Protein-coding
8_BMSC_peak_101958_lociStitched	Chr7	112973906	113001251	27345	RAT17	ncRNA

**Table 6:** Detailed information of super enhancers. D14 group.

ID	Chrom	Start	End	Size	Target gene	Gene type
2_osteoblast_peak_1318_lociStitched	Chr10	90674066	90676304	2238	LOC101926942	ncRNA
2_osteoblast_peak_3420_lociStitched	Chr15	89119260	89121050	1790	ABHD2	Protein-coding
2_osteoblast_peak_6765_lociStitched	Chr4	90317314	90319003	1689	CCSER1	Protein-coding
2_osteoblast_peak_8606_lociStitched	Chr7	18638278	18640106	1828	HDAC9	Protein-coding

**Table 7:** The super enhancer target gene expression changes during osteogenesis of hBMSCs.

Super enhancer target gene	D0	D14
LINC00460	1.08 ± 0.06	0.54 ± 0.04
LINC00844	0.97 ± 0.02	0.11 ± 0.01
KCNMA1-AS1	1.04 ± 0.03	5.72 ± 0.52
ASTN2-AS1	1.12 ± 0.08	1.44 ± 0.12

## Data Availability

The data used to support the findings of this study are available from the corresponding author upon request.

## Abbreviations

SEs: Super enhancers
hBMSCs: Human bone marrow mesenchymal stem cells
TGF-*β*: Transforming growth factor *β*
PI3K: Phosphoinositide 3-kinase
ECM: Extracellular matrix
RT-qPCR: Real-time fluorescence quantitative polymerase chain reaction
TEs: Typical enhancers
WB: Western blot
RUNX2: Runt-related transcription factor 2
OPN: Osteopontin
COL1A1: Collagen type I alpha 1
ChIP-seq: Chromatin immunoprecipitation-sequencing
MACS: Model-based analysis of ChIP-seq
GO: Gene ontology
DAVID: Database for annotation, visualization, and integrated discovery
KEGG: Kyoto encyclopedia of genes and genomes
MF: Molecular functions
CC: Cell composition
BP: Biological processes
mTFs: Master transcription factors
C/EBP-*α*: CCAAT enhancer-binding protein alpha
Med1: Mediator complex subunit 1
MAPK: Mitogen-activated protein kinase
NF-*κ*B: Nuclear factor kappa B
FGF: Fibroblast growth factor
BMPs: Bone morphogenetic proteins
SMADs: Drosophila mothers against decapentaplegic protein
STAT1: Signal transducer and activator of transcription 1
PKC: Protein kinase C
LncRNA: Long noncoding RNA
miRNA: Micro RNA.
